The article "Exploratory Study on Expression of Fatty Tissue in Gestational Diabetes Mouse" was retracted in 2023. Reasons: unreliable results or conclusions; concerns about the data; concerns about the peer review; concerns about the citations.

# Exploratory Study on Expression of Fatty Tissue in Gestational Diabetes Mouse

**DOI:** 10.1155/2021/6813147

**Published:** 2021-10-05

**Authors:** Xiaoling Zhou, Xin Li, Tingting Wei, Ying Xu, Yunyuan Mao, Chen Lei

**Affiliations:** ^1^Department of Nephrology, General Hospital of Ningxia Medical University, Yinchuan, Ningxia 750004, China; ^2^Department of Endocrinology, General Hospital of Ningxia Medical University, Yinchuan, Ningxia 750004, China; ^3^Department of Geriatrics and Special Needs, General Hospital of Ningxia Medical University, Yinchuan, Ningxia 750004, China

## Abstract

**Objective:**

To investigate the changes of UCP1 protein in brown fat by establishing a model of gestational diabetes mellitus through intervention of high fat and carbohydrate diet. To explore the changes of UCP1 protein in brown fat in gestational diabetic mice, and analyze the characteristics of abnormal glucose metabolism in gestational diabetic mice and its relationship with changes in adipocyte morphology and insulin resistance.

**Methods:**

Eighty C57BL/6J pregnant mice were randomly divided into a normal control group and a high-fat and high-sugar feeding group. The normal control group was fed a normal diet, while the high-fat and high-sugar group was fed a high-fat and high-sugar diet to establish a gestational diabetes mellitus (GDM) model. On the pregnancy days 0, 10, and 18, the weight and fasting glucose were measured. On the pregnancy day 18, the triglycerides (TG), the total cholesterol (TC), free fatty acid (FFA), insulin levels, and insulin resistance index (HOMA-IR) were measured or calculated. At the same time, brown fat UCP1 protein of the two groups of pregnant mice were measured using Western blot Observed the Adipose tissue pathological changes by staining HE. The adipocyte was observed, and the correlation was analyzed.

**Results:**

Twenty-one pregnant mice reach the level of gestational diabetes diagnosis (FBG ≥ 5.1 mmol/L) in the high-fat and high-sugar diet group. On the pregnancy day 10 and 18, the fasting plasma glucose and the body weight significantly increased (*P* < 0.05). The total cholesterol, triglycerides, free fatty acid, insulin level, and insulin resistance index of the GDM group were also higher compared with that of the control group (*P* < 0.05). The adipocyte size significantly increased in the GDM mice. TG, TC, FFA, and body weight at 18 days of gestation were significantly correlated with HOMA-IR and single-adipocyte area in the GDM mice. HOMA-IR was significantly correlated with a single-adipocyte area. Compared with the normal control group, the UCP1 proteins of GDM mice decreased significantly and negatively correlated with body weight increase.

The article "Exploratory Study on Expression of Fatty Tissue in Gestational Diabetes Mouse" was retracted in 2023. Reasons: unreliable results or conclusions; concerns about the data; concerns about the peer review; concerns about the citations.

**Conclusion:**

Feeding C57BL/6J pregnant mice with high fat and high sugar to establish a gestational diabetes mouse model has good stability and is similar to human gestational diabetes. The reduction of brown fat UCP1 protein in GDM mice has a certain correlation with obesity tendency and obvious insulin resistance.

## 1. Introduction

Diabetes mellitus is a syndrome of metabolic disorders of various substances characterized by chronic elevated blood glucose levels due to deficiencies in insulin secretion and/or action caused by various etiologies and pathogenic factors [1]. Usually, this disease is caused by defective secretion of insulin and/or defective action of insulin. Pregnancy is a special period of human beings; the body is in a state of stress at this time; and the various organs of the body will occur a series of endocrine metabolic disorders, of which carbohydrate and lipid metabolic disorders are an important factor leading to the onset of gestational diabetes mellitus (GDM). Usually, there are two combinations of gestational status and diabetes mellitus. The first is that pregnant women have been clearly diagnosed with diabetes before pregnancy and continue to have diabetes mellitus after the birth of the fetus, which is called pregnancy with diabetes mellitus; the other is GDM, which is abnormal blood sugar metabolism first found or occurred during pregnancy. According to the latest diagnostic criteria, the global incidence of gestational diabetes accounts for 17.8% of pregnant women [2]. The incidence of GDM varies from country to country in the world. At present, the reported incidence is 1.7%–11.6% [3]. The incidence of GDM in China is about 1.2%; among them, more than 80% of patients had first found diabetes during pregnancy, and less than 20% of patients had diagnosed diabetes mellitus before pregnancy [4]. At present, the etiology of GDM is not very clear; it is believed that it is mainly related to insulin resistance, insulin secretion deficiency, autoimmunity, heredity, and other factors [5]. During pregnancy, the sensitivity of the surrounding tissues to insulin decreases with the increase in gestational weeks, resulting in so-called insulin resistance. Recent studies have shown that besides the above reasons, the occurrence of GDM is also related to the rapid growth of body weight during pregnancy, the secretion of adipocytokines, the release of inflammatory factors, genetic genes, natural and social environment, and other factors [6]. In order to maintain normal glucose metabolism during pregnancy, insulin beta cells must produce 2–5 times or more insulin under normal conditions in order to counteract the effect of insulin resistance and maintain the dynamic balance of normal glucose metabolism [7]. After 24 weeks of gestation, the body's “insulin resistance” begins to increase. If the insulin secretion function of islet beta cells is reduced at this time, it cannot compensate for the absolute insulin dosage caused by insulin resistance. Or when the blood sugar is relatively insufficient, it begins to rise continuously at this time, which will lead to the occurrence of high blood sugar. At present, the incidence of diabetes is on the rise in the world. It is predicted that the number of diabetes patients will reach 438 million by 2020, while Asian patients will account for nearly half of the total. Diabetes will be the leading cause of death in most developed countries [8].

The article "Exploratory Study on Expression of Fatty Tissue in Gestational Diabetes Mouse" was retracted in 2023. Reasons: unreliable results or conclusions; concerns about the data; concerns about the peer review; concerns about the citations.

Recent studies have shown that besides normal physiological insulin resistance, GDM patients also have pathological insulin resistance, which is closely related to the cytokines associated with insulin resistance (IR). In recent years, more and more studies have shown that adipose tissue is the starting site of insulin resistance. When metabolic changes and external stimulation occur, adipose tissue can secrete a variety of physiologically active proteins, also known as adipocytokines, including free fatty acids (FFA) [9], leptin (LEP) [10], and tumor necrosis factor-alpha (TNF-alpha) [11], plasminogen activator inhibitor-1 (PAI-1), resistin (RETN), and adiponectin (ADPN) [12] can participate in complex physiological and pathological processes. White fat is a major organ of energy storage in mammals, and it regulates whole-body metabolism and increases insulin resistance by releasing hormones and cytokines. In obesity, the volume and number of white adipocytes increased. On the contrary, brown fat plays an important role in energy consumption [13]. Its main function is to participate in fatty acid oxidation. The energy produced is released by uncoupling protein (UCPs) to heat energy, which promotes energy metabolism and consumption, and increases insulin sensitivity and weight loss. Insulin resistance index was negatively correlated with brown fat, that is, the higher the brown fat content, the smaller the insulin resistance coefficient [14].

The commonly used models of GDM are divided into spontaneous animal models and induced or experimental animal models. Spontaneous animal models have reduced human factors, and the pathogenesis of some diseases is consistent with human diseases. It is an ideal animal model. But this kind of laboratory animal is expensive and very limited. Experimental animal models can be used to induce disease models in a short time by strictly controlling various restrictive conditions, so as to achieve the purpose and requirement of research. At present, there are three ways of experimental animal models of gestational diabetes in the world: chemical drug induction, diet induction, and surgery induction. Among them, the experimental models induced by streptozotocin (STZ) and other drugs can directly damage pancreatic function, lead to hyperglycemia or instability, and limit the credibility of the results [15, 16]. The simple high-fat diet induction model, which has the closest pathogenesis to human clinical GDM, avoids direct damage to organ function and has certain rationality for the study of GDM [17]. Heterozygous C57BL mice are mutant with an ob/ob genetic background. Leptin gene mutation in this mouse resulted in leptin deficiency. Studies have proved that the metabolism of this kind of mice is slow, and a high-fat and high-sugar diet can quickly and effectively induce the increase of blood sugar, which is similar to the metabolic characteristics of human metabolic diseases. Some models of gestational diabetes animal models have been reported at home and abroad. However, there are no mature animal models for gestational diabetes in many animal laboratories in China. The animal model of GDM was prepared from the metabolic characteristics of C57BL mice, the special pathophysiological changes during pregnancy, and the induction of high fat and high carbohydrate diet.

The article "Exploratory Study on Expression of Fatty Tissue in Gestational Diabetes Mouse" was retracted in 2023. Reasons: unreliable results or conclusions; concerns about the data; concerns about the peer review; concerns about the citations.

At present, there are many studies on the pathogenesis and related factors of GDM, but the relationship with UCPs is not very clear. Studies have shown that phycophaein can reduce obesity induced by high-fat and high-sugar diet by increasing uncoupling protein 1 (UCP1) in brown fat of rats. In the enhanced expression group of UCP1, body weight was significantly reduced, and insulin sensitivity was significantly increased. In this study, the model of GDM mice was established by high-fat and high-sugar diet induction. The changes of UCP1 protein in fat brown fat of GDM mice and non-GDM mice, the metabolism of sugar and lipid, and the relationship between the morphological changes of adipocytes and insulin resistance in gestational diabetic mice were investigated.

## 2. Research Design and Methods

### 2.1. Animals

100 healthy and clean C57BL / 6J female mice and 40 male mice, 8 weeks old, weighing 20–25 g, were provided by Weitong Lihua Experimental Animal Technology Co., Ltd. The feed for ordinary laboratory animals was provided by Beijing Keao Xieli Feed Co., Ltd. The mice in the experiment were placed in the feeding room with the temperature of 22–26°C, the air unblocked, and the relative humidity of 40%–70%. Female and male mice were fed in separate cages, fed freely with water, and replaced with padding regularly.

The article "Exploratory Study on Expression of Fatty Tissue in Gestational Diabetes Mouse" was retracted in 2023. Reasons: unreliable results or conclusions; concerns about the data; concerns about the peer review; concerns about the citations.

### 2.2. Grouping and Model Making of Experimental Animals

All male and female mice were fed with normal laboratory animal feed for two weeks. Then the male and female mice were caged at 2:1 at 5 p.m., and the vaginal emboli or vaginal secretions were examined by microscopy at 9 a.m. If sperm or vaginal embolus is found under a microscope, pregnancy can be considered, and the gestational age is calculated by recording the gestational day as 0 days. If the female rat is not pregnant, it will continue to cage with the male, and the female rat that is not pregnant for a week will be abandoned. During the experiment, 80 mice successfully became pregnant, and 20 mice were abandoned. The pregnant mice were fed separately and randomly divided into two groups: normal feed group (40 mice) and high-fat and high-sugar feed group (40 mice). The two groups were fed with common feed and high-fat and high-sugar feed, respectively, and were fed with water freely. All pregnant mice were randomly divided into two groups according to the random number table: the normal diet group and the high-fat and high-sugar diet group. Common feed is full nutrition feed. High-fat and high-sugar feed adds 15% lard, 10% yolk, and 10% sugar on the basis of 65% common feed. At present, there is no unified diagnostic standard for GDM in mice. According to the seminar of experts, the diagnosis of GDM can be diagnosed if the fasting blood glucose is more than 5.1 mmol/L [18]. Therefore, according to the blood glucose diagnostic criteria of GDM, we set the model of GDM as the diagnostic criteria of GDM in mice with fasting blood glucose in the middle and late pregnancy, as well as fasting blood glucose in the 18th day (≥5.1 mmol/L). The levels of fasting blood glucose (FPG), insulin (FINS), and insulin resistance index (IR) were significantly increased, suggesting that pregnant mice fed with high-fat and high-sugar diet conformed to the characteristics of pathological IR in GDM patients.

### 2.3. Specimen Collection

On day 0 of gestation, the mice were subtracted from the tip of the tail by about 2 mm, and the blood was dripped on the blood sugar test paper to measure the fasting blood sugar. After fasting for 12 hours, mice were anesthetized on the 18th day and took blood from eyeballs. After fixed experimental animals were anesthetized, the skin was disinfected with 75% of the medical alcohol. The T was cut along the middle of the abdomen (to the plane of the diaphragm). Offspring mice are taken out and weighed. The extraperitoneal fat tissue of the pregnant mice was removed and placed in the centrifuge tube. The number was marked and recorded, then stored in the −80 C refrigerator. This research was approved by the medical ethics committee of General Hospital of Ningxia Medical University (AEE18069). The killing process of all mice complied with relevant regulations and did not increase pain.

The article "Exploratory Study on Expression of Fatty Tissue in Gestational Diabetes Mouse" was retracted in 2023. Reasons: unreliable results or conclusions; concerns about the data; concerns about the peer review; concerns about the citations.

### 2.4. Observation and Monitoring Indicators

The changes in urine and water intake were observed every day. Electronic scales were used to weigh at 0 and 18 days of gestation. After fasting, blood samples were taken from the tail of pregnant mice with tissue scissors, and fasting blood sugar was measured with blood glucose test paper and blood glucose meter (Roche Vigor, Germany). Fasting insulin, cholesterol, triglyceride, and FFA acid were detected by ELISA. The kidneys were removed for 10% formaldehyde solution and fixed for 24 hours, and the thickness of tissue blocks was about 0.5 cm. Routine dehydration, transparency, wax impregnation, embedding, slicing (thickness 5 *μ*m), and hematoxylin eosin (HE) staining were performed to count the number of fat cells in a single visual field (20 × 10), and the average area of the total adipose cell (total area/total cell number) was calculated. The total area of a single 20*∗*10-fold field of vision is 39,970 *μ*m^2^.

### 2.5. Western Blotting Analysis

Samples of extraperitoneal adipose tissue from pregnant mice were collected on the 18th day of pregnancy and stored at −80°C until use. For total protein extraction, protein concentration was measured using Pierce BCA Protein Assay Kit. The proteins were separated on SDS-PAGE and transferred to the PVDF membrane using Trans-Blot Turbo semidry transfer system (Bio-Rad). The membrane was incubated with the following primary antibodies (UCP1, 1:1000; *β*-action, 1:1000) from cell signaling technology diluted in blocking buffer overnight at 4°C. Normalization of the signals was done using REVERT total protein stain (LI-COR). PVDF film was placed in SuperSingal chemiluminescent reagent for 2 minutes. BiospectrumAC gel imaging analysis system was used to scan and save the analysis pictures.

### 2.6. Statistical Methods

Statistical package for the social sciences (SPSS) 19.0 was used for statistical analysis. The results of all data were expressed as mean ± standard deviation ($\bar{x}$ ± *s*). The comparison between the two groups was performed by *t*-test, *P* < 0.05 being statistically significant.

## 3. Results

### 3.1. Modeling of GDM Mice

Twenty-one of the 40 pregnant mice in the high-fat and high-sugar died group had fasting blood sugar (≥5.1 mmol/L), which met the diagnostic criteria for GDM. Eight of the 40 pregnant mice in the normal diet group had elevated blood sugar, which was excluded from the normal control group. Thirty-two mice with stable blood sugar were included in the normal control group.

The article "Exploratory Study on Expression of Fatty Tissue in Gestational Diabetes Mouse" was retracted in 2023. Reasons: unreliable results or conclusions; concerns about the data; concerns about the peer review; concerns about the citations.

### 3.2. Observation of General Conditions of Mice and Their Offspring in Each Group

The amniotic fluid was clear, and the placenta was bright red in the normal control group. There was no bleeding and the development of offspring was basically normal. The amniotic fluid in the GDM group was turbid; the placenta was darker; the body weight of offspring was larger than that of the normal control group; and one of them had developmental abnormalities such as stillbirth.

### 3.3. General Changes of Pregnant Mice in Each Group

The weight of pregnant mice in each group on day 0, 10, and 18 was weighed by electronic weighing. The weight of pregnant mice on day 10 and 18 of GDM mice was significantly higher than that of the normal control group (*P* < 0.05). There was statistical significance (Table 1 and Figure 1). The fasting blood glucose of pregnant mice in different periods was measured by tail blood collection. We found that the blood glucose of pregnant GDM mice on the 10th and 18th day of gestation was significantly higher than that of the normal control group (*P* < 0.05; Table 1; Figure 2).

### 3.4. Changes of Fasting Insulin Level, Insulin Resistance, Serum Triglyceride, Total Cholesterol, and Free Fat in Pregnant Mice

The levels of FINS, insulin resistance (HOMA-IR), triglyceride (TG), total cholesterol (TC), and FFA in gestational diabetic mice on day 18 were significantly higher than those in the normal control group (*P* < 0.05; Table 2).

### 3.5. Pathological Observation of Adipose Tissue in Each Group

Table 3 showed that the number of adipocytes in the gestational diabetes group was significantly lower than that in the normal control group (*P* < 0.05) under the same magnification microscope (Figure 3), and the single-adipocyte area was significantly larger than that in the normal control group (*P* < 0.05; Figure 4).

### 3.6. Correlation Analysis of Serum Triglyceride, Total Cholesterol, Free Fatty Acid, and Body Weight of Pregnant Mice at 18 Days with Insulin Resistance and Single-Adipocyte Area

The data showed that TG, TC, FFA, and body weight at 18 days of gestation were significantly correlated with HOMA-IR and single-adipocyte area (*P* < 0.001), and there was a positive correlation between them, as shown in Table 4 and Figures 5–14.

### 3.7. The Expression of UCP1 Protein in Normal and GDM Groups

Western blot analysis showed that the expression of UCP1 protein in the GDM group was significantly lower than that in the normal control group (Figure 15).

## 4. Discussion

GDM (GDM) refers to abnormal glycometabolism first found or occurred during pregnancy. Insulin resistance plays a major role in the pathogenesis of gestational diabetes. During normal pregnancy, the secretion of hormones in the body of pregnant women increases significantly during pregnancy. Such as glucocorticoid, progesterone, placental prolactin, prolactin, estrogen, and progesterone, which are the insulin antagonist hormones, resulting in their insulin resistance, belonging to normal physiological insulin resistance. With the progress of pregnancy cycle, insulin resistance gradually increased and reached its peak in the third trimester of pregnancy. When insulin secretion of islet beta cells cannot meet the body's demand for insulin and insulin resistance loss, it leads to glucose metabolism disorders in some pregnant women and then to GDM. Recent studies have shown that in addition to normal physiological insulin resistance, patients with GDM (GDM) also have pathological insulin resistance, which is closely related to the cytokines associated with insulin resistance (IR). In recent years, more and more studies have shown that adipose tissue is the starting site of insulin resistance. When metabolic changes and external stimulation occur, adipose tissue can secrete a variety of physiologically active proteins, also known as adipocytokines, including free fatty acid (FFA), leptin (LEP), tumor necrosis factor alpha (TNF-alpha), plasminogen activator inhibitor-1 (PAI-1), interleukin-6 (IL-6), resistin (RETN), adiponectin (ADPN), and so on can participate in complex physiological and pathological processes.

The article "Exploratory Study on Expression of Fatty Tissue in Gestational Diabetes Mouse" was retracted in 2023. Reasons: unreliable results or conclusions; concerns about the data; concerns about the peer review; concerns about the citations.

In the third trimester of pregnancy (about 18 days of gestation), it showed that the drinking water consumption of the GDM group was faster than that of the normal control group, and the two groups of pregnant mice changed the padding at the same time. The gestational diabetes group was obviously wet. On the 18th day of gestation, the body weight and fasting blood glucose of the GDM group increased significantly compared with the normal control group (*P* < 0.05), and the clinical manifestations of polydipsia, polyphagia, and polyuria in the GDM group were consistent with the clinical characteristics of diabetes mellitus. This suggests that a high-fat diet can induce obesity in C57BL/6J mice in a short period of time, and a high-fat and high-sugar diet can exacerbate the rapid rise of fasting blood sugar in pregnancy. The determination of triglyceride, cholesterol, and free fatty acid showed that the TC, TG, and FAA of pregnant mice in the GDM group were significantly higher than those in the normal control group, and the difference was statistically significant (*P* < 0.05), indicating that high-fat and high-sugar diet could increase triglyceride, cholesterol, and free fatty acid.

The article "Exploratory Study on Expression of Fatty Tissue in Gestational Diabetes Mouse" was retracted in 2023. Reasons: unreliable results or conclusions; concerns about the data; concerns about the peer review; concerns about the citations.

The serum insulin level in the GDM group was significantly higher than that in the normal control group (*P* < 0.05), which indicated that a high-sugar and high-fat diet could stimulate the islet beta cells of pregnant mice to increase insulin secretion, and the insulin resistance index in the GDM group was significantly higher than that in the normal control group, which indicated that the difference was statistically significant (*P* < 0.05). A high-fat and high-sugar diet can significantly aggravate insulin resistance in pregnant mice.

There is a general insulin resistance during pregnancy, which leads to the increase of insulin level, will appear physiological insulin resistance. The blood insulin level of GDM patients is higher; insulin resistance is more serious than a normal pregnancy; and pathological insulin resistance appears, which shows the clinical characteristics of diabetes mellitus. Because insulin resistance occurs in GDM, islet beta cells secrete a large amount of insulin compensatively, and the body is in a state of high insulin. Insulin can transport glucose to cells by promoting glucose carriers in muscle and adipose tissue cells, providing the necessary glycerol and fatty acids for the synthesis of triglycerides, promoting fat synthesis and storage, and reducing blood-free fat. At the same time, through inhibiting hormone-sensitive lipase in adipose tissue and the decomposition and oxidation of fat in adipocytes, the rate of fat mobilization can be slowed down, and fat accumulation can be further promoted. Therefore, body fat metabolism is vigorous; blood lipid is elevated; hyperlipidemia occurs; and then a series of pathological changes in tissues and organs occur. GDM animal model is simulated in the late pregnancy in a pathological insulin resistance state; the body secreted a lot of insulin, increased the accumulation of body fat, and formed a vicious circle between insulin resistance and hyperlipidemia.

With the deepening of the research on GDM, the changes of body metabolism during GDM cannot be ignored. In addition to abnormal glucose metabolism, GDM patients also have abnormal lipid metabolism in varying degrees. Due to the particularity of pregnancy, the mother needs to take in a large amount of lipid nutrients to meet the needs of the mother itself and the normal development of the fetus. The blood lipid level of normal pregnant women will also increase with the increase of gestational weeks. In the third triglyceride, cholesterol and other blood lipid indicators are significantly higher than those of non-pregnant women. Because human placental prolactin and blood lipid increase with the increase of gestational weeks, these changes are consistent with the increase of fat nutrients intake by pregnant women in order to meet the needs of normal fetal development [11, 12]. There is no pathological significance for the increase of blood lipid in normal pregnancy to be physiological hyperlipidemia. The level of blood lipid increases with the aggravation of abnormal glucose metabolism. Because of the pathological insulin resistance and abnormal glucose metabolism, the increase of blood lipids will be more obvious. The disorder of lipid metabolism has become one of the pathophysiological characteristics of GDM. Previous studies have shown that TG, very low-density lipoprotein cholesterol (VLDL-c), low-density lipoprotein cholesterol (LDL-c), and high-density lipoprotein cholesterol (HDL-C) in normal pregnant women are higher than those in healthy non-pregnant women. The serum lipid level reaches its peak in the third trimester of pregnancy and returns to normal gradually after delivery. This may be due to the adaptive change of maintaining normal growth and development of the fetus during pregnancy. It may also be due to increased intestinal fat absorption during pregnancy, as well as the combined effects of progestational hormone (PRH) and human placental lactogen (HPL) and other factors causing insulin resistance [19].

The article "Exploratory Study on Expression of Fatty Tissue in Gestational Diabetes Mouse" was retracted in 2023. Reasons: unreliable results or conclusions; concerns about the data; concerns about the peer review; concerns about the citations.

In this study, diabetic pregnant mice induced by high-fat and high-sugar diet showed an abnormal increase in blood sugar and lipid (triglyceride and cholesterol) in the third trimester of pregnancy, and insulin resistance also existed. This is consistent with abnormal blood sugar and lipid in human pregnancy. The increase of blood sugar and blood lipid was more obvious in GDM pregnant mice, and there was pathological insulin resistance, which further stimulated insulin secretion by islet beta cells and aggravated the abnormal lipid metabolism. It further shows that human GDM can also have abnormal blood sugar and lipid levels, and there is pathological insulin resistance. Studies have shown that the size of adipocytes is an important determinant of the synthesis of cytokines. Hypertrophy of adipocytes reduces the relative supply of blood, leading to disorders in cell function [20]. Macrophages in adipose tissue ingest fat and secrete a variety of inflammatory factors, acting together with adipocytokines secreted by themselves on insulin target cells, activating chronic inflammatory response, and blocking insulin receptor signaling pathway, thus causing insulin resistance [21]. In this experiment, the high-fat and high-sugar diet-induced diabetic mice group, GDM adipose tissue pathological section showed that the number of adipocytes in the gestational diabetes group was significantly less than that in the normal control group (*P* < 0.05) under the same magnification microscope, and the area of single fat cells was significantly larger than that in the normal control group (*P* < 0.05).

The article "Exploratory Study on Expression of Fatty Tissue in Gestational Diabetes Mouse" was retracted in 2023. Reasons: unreliable results or conclusions; concerns about the data; concerns about the peer review; concerns about the citations.

Pregnant women often eat too much high-fat and high-sugar food during pregnancy, which leads to fat accumulation in the body and excessive lipid storage in adipocytes leading to adipocyte enlargement and dysfunction. Due to the increased insulin resistance in GDM, the sensitivity of insulin receptors distributed on the surface of adipocyte membrane to insulin decreases greatly, resulting in the antilipid effect of adipocytes be weaken. A large number of fatty acids are released from adipocytes into the blood, providing raw materials for the synthesis of triglycerides; secondly, because the activity of insulin resistance lipoprotein esterase decreases greatly, low- to high-density lipoprotein conversion ability also decreased, high-density lipoprotein production increased, and low-density lipoprotein apolipoprotein glycosylation also reduced the decomposition of low-density lipoprotein; increased free fatty acid (FFA) has competitive inhibition on the aerobic oxidation and anaerobic hydrolysis of sugar. Studies have shown that high levels of free fatty acids can inhibit the use of sugar in muscle tissue and liver and impair the function of islet cells, while reducing the sensitivity of insulin receptors and increasing insulin resistance [22]. The decreased sensitivity of islet beta cells to glucose and the increased resistance of peripheral tissues to insulin in GDM make islet beta cells secrete more insulin compensatively, thus increasing the workload of islet beta cells, accelerating the proliferation and functional failure of islet beta cells, and increasing the risk of type 2 diabetes mellitus after pregnancy.

Uncoupling protein 1 is a transporter that regulates proton transmembrane transport and enhances resting metabolic rate. UCP1 protein has been reported to increase insulin sensitivity [23]. UCP1 is mainly distributed in brown adipose tissue (BAT), and brown adipose tissue is the main heat-producing tissue. Uncoupling protein 1 is associated with obesity in rodents. Obesity and diabetes can occur in genetically modified mice that artificially cause uncoupling protein 1 deficiency or remove brown fat. The AG variant of UCP1 and the beta 3 adrenergic receptor Trp64Arg polymorphism may have a synergistic effect on weight gain. UCP1 is expressed only in brown adipose tissue (BAT). UCP1 is a protein encoded by the UCP1 gene containing 306 amino acids, consisting of 6C or N ends toward the transmembrane region of the cytosol. UCP1 is homologous to ADP/ATP vector, and its activity is inhibited by purine nucleotides. UCP1 can transport fatty acid anions from the inner surface of the mitochondrial inner membrane to the outer surface, protonate the anions on the outer surface, change the charge to neutral, and then return to the inner surface of the mitochondrial inner membrane. This process promotes proton transport to the mitochondrial inner membrane, reduces proton electrochemical potential gradient, and decouples oxidative phosphorylation and ATP synthesis. Therefore, the role of UCP1 is to increase energy consumption and heat production. In this experiment, we detected UCP1 protein in adipose tissue of GDM and normal control group and found that the expression of UCP1 in the gestational diabetes group was significantly lower than that in the normal control group.

The article "Exploratory Study on Expression of Fatty Tissue in Gestational Diabetes Mouse" was retracted in 2023. Reasons: unreliable results or conclusions; concerns about the data; concerns about the peer review; concerns about the citations.

To sum up, this experiment establishes a gestational diabetes mouse model by high-fat and high-sugar diet induction method, which can well simulate the pathogenesis of GDM in the human body, and the model shows that GDM not only has abnormal glucose metabolism but also has abnormal lipid metabolism. Through the detection of blood glucose and blood lipids, it was found that blood glucose and blood lipid levels increased significantly. Through pathological observation of adipose tissue, it was found that the number of adipocytes in the gestational diabetes group was significantly lower than that in the normal control group under the same magnification microscope, and the single-adipocyte area was significantly larger than that in the normal control group, and there was obvious insulin resistance. By detecting the UCP1 protein, it was found that the expression of UCP1 protein in the gestational diabetes group was significantly lower than that in the normal control group, indicating that there was a certain correlation between the UCP1 protein and the occurrence of GDM, and it is negatively correlated.

## 5. Conclusions

1. The establishment of the gestational diabetes model in pregnant mice induced by a high-fat and high-sugar diet is closer to the pathogenesis of human GDM, and the model is more stable.
2. The decrease of UCP1 protein in brown fat is related to the incidence of gestational diabetes.
3. Obesity in gestational diabetic mice is prone to occur and has obvious insulin resistance.
4. Fasting insulin, insulin resistance, serum triglyceride, total cholesterol, and free fat in group GDM were higher than those in the normal control group.
5. The adipocytes of GDM mice were significantly larger than those of the normal control group.

The article "Exploratory Study on Expression of Fatty Tissue in Gestational Diabetes Mouse" was retracted in 2023. Reasons: unreliable results or conclusions; concerns about the data; concerns about the peer review; concerns about the citations.

## Figures and Tables

**Figure 1:** The weight change of pregnant mice in each group.

**Figure 2:** Changes of fasting blood glucose in different periods of pregnant mice in each group.

**Figure 3:** Number of fat cells in pregnant mice in each group.

**Figure 4:** The area of a single fat cell in each group of pregnant mice.

**Figure 5:** HE staining of adipose tissue of pregnant mice in each group.

**Figure 6:** Correlation analysis between HOMA-IR and TC.

**Figure 7:** Correlation analysis between HOMA-IR and TG.

**Figure 8:** Correlation analysis between HOMA-IR and FFA.

**Figure 9:** Correlation analysis between HOMA-IR and 18 d BW.

**Figure 10:** Correlation analysis between HOMA-IR and single-cell area.

**Figure 11:** Correlation analysis between TC and single-cell area.

**Figure 12:** Correlation analysis between TG and single-cell area.

**Figure 13:** Correlation analysis between 18 d BW and single-adipocyte area.

**Figure 14:** Correlation analysis between FFA and single-adipocyte area.

**Figure 15:** The expression of UCP1 protein in normal and GDM.

**Table 1:** Comparison of the changes of body weight and blood sugar in different gestational weeks.

Data	Normal (*n* = 32)	GDM (*n* = 21)
0 d BW (g)	21.68 ± 0.71	22.35 ± 1.28
10 d BW (g)	27.53 ± 1.14	30.30 ± 2.54^*∗*^
18 d BW (g)	35.19 ± 1.56	41.83 ± 2.33^*∗*^
0 d Glu (mmol/L)	4.72 ± 0.31	4.93 ± 0.46
10 d Glu (mmol/L)	4.11 ± 0.29	5.51 ± 0.22^*∗*^
18 d Glu (mmol/L)	3.80 ± 0.31	5.73 ± 0.31^*∗*^

*Note.P* < 0.05.

**Table 2:** Comparison of insulin resistance, insulin level, triglyceride, total cholesterol, and free fatty acids in different groups.

Data	Normal (*n* = 32)	GDM (*n* = 21)
FINS (mIU/L)	19.21 ± 0.69	21.48 ± 2.87^*∗*^
HOMA-IR	3.79 ± 0.21	5.95 ± 0.86^*∗*^
TC (mg/dL)	42.74 ± 9.18	60.11 ± 9.95^*∗*^
TG (mg/dL)	47.92 ± 4.01	63.79 ± 5.42^*∗*^
FFA (mmol/L)	0.31 ± 0.01	0.44 ± 0.02^*∗*^

*Note*. *P* < 0.05.

**Table 3:** Number and area of cells in a single field of vision.

Data	*n*	Number	Single-adipocyte area (*μ*m^2^)
Normal	32	120.63 ± 1.08	2659.33 ± 25.24
GDM	21	97.71 ± 0.83^*∗*^	3279.32 ± 28.11^*∗*^

*Note.P* < 0.05.

**Table 4:** Correlation analysis of triglyceride, total cholesterol, free fatty acid, and body weight of pregnant mice at 18 days with insulin resistance and single-adipocyte area.

Data		Area	HOMA-IR	TG	TC	FFA	18 d BW
HOMA-IR	*R*	0.774^*∗*^	1.000	0.793^*∗*^	0.756^*∗*^	0.833^*∗*^	0.799^*∗*^
Area	*r*	1.000	0.774^*∗*^	0.752^*∗*^	0.598^*∗*^	0.693^*∗*^	0.801^*∗*^

*Note.P* < 0.001.

## Data Availability

The data can be obtained from the corresponding author upon reasonable request.
